RETRACTED

# Hypoxia-Induced Nestin Regulates Viability and Metabolism of Lung Cancer by Targeting Transcriptional Factor Nrf2, STAT3, and SOX2

**DOI:** 10.1155/2022/9811905

**Published:** 2022-08-30

**Authors:** Yongshi Liu, Xinglin Zhang, Tao Jiang, Ning Du

**Affiliations:** ^1^Department of Thoracic Surgery, Tangdu Hospital, Air Force Medical University, Xi'an, Shaanxi, China; ^2^Department of Oncology, Qingdao Municipal Hospital, Qingdao, Shandong, China; ^3^Department of Thoracic Surgery, The First Affiliated Hospital of Xi'an Jiaotong University, Xi'an, Shaanxi, China

## Abstract

**Objective:**

To investigate hypoxia-induced Nestin regulates lung cancer viability and metabolism by targeting transcription factors Nrf2, STAT3, and SOX2.

**Methods:**

Eighty-four cases of nonsmall cell lung cancer (nonsmall cell lung cancer, NSCLC), which had been treated from June 2020 to February 2021, were randomly selected from our clinicopathology database. Immunohistochemical staining of collected tissue cells was performed to assess the expression patterns of Nestin, STAT3, Nrf2, and SOX2. Data were quantified and statistically analyzed using one-way and two-way ANOVA tests with *P* < 0.05.

**Results:**

Clinicopathological findings showed significant differences in lymph node metastasis, tissue differentiation, and histology on induction of Nestin expression; Nestin expression correlated with STAT3, Nrf2, and SOX2 expression.Nestin/STAT3/SOX2/Nrf2 are involved in angiogenesis and lung cancer development.

**Conclusion:**

Hypoxia-induced Nestin promotes the progression of nonsmall lung cancer cells by targeting the downstream transcription factors STAT3, Nrf2, and SOX2.

## 1. Introduction

According to the Global Cancer Survey, approximately 1.8 million people will die from lung cancer in 2020 [1]. Primary bronchial lung cancer is currently the fastest growing tumor in terms of incidence and mortality, and it is clinically classified into small cell lung cancer (SCLC) and nonsmall cell lung cancer (NSCLC) according to the pathological pattern, of which NSCLC accounts for about 80% of the total incidence of lung cancer. NSCLC accounts for about 80% of the total incidence of lung cancer, and the symptoms of NSCLC invasion and metastasis have received more and more attention and research in recent years [2]. Compared with SCLC, NSCLC is relatively slow to spread and metastasize, but most patients already have organ metastasis at the time of diagnosis and are prone to irreversible migration to bone and central nervous system, resulting in poor prognosis and reduced 5-year survival rate of NSCLC patients [3]. The transcription factors Nrf2, STAT3, and SOX2 are multifunctional proteins [4], and several studies have shown that the abnormal expression of Nrf2, STAT3, and SOX2 can play a regulatory role in tumor proliferation and metastasis by interacting with different protein cofactors, including NSCLC, however, the role of Nrf2, STAT3, and SOX2 in NSCLC is still not well studied. The mechanisms of Nrf2, STAT3, and SOX2 in NSCLC are not well studied, and further research is needed.

RETRACTED

Nestin is a plastic cytoskeletal protein whose expression may vary with the functional state of the cell and is widely used as a marker for neuronal cells derived from embryonic stem cells (hES cells) and induced pluripotent stem cells (iPS cells). Nestin expression in tumor cells has been reported to result in chemoresistance in hepatocellular carcinoma cell lines and radioresistance in nasopharyngeal carcinoma cell lines [5, 6]. Previously, Nestin has been reported to be associated with neuroendocrine features and involved in malignant phenotypes including cell growth. Other investigations have also shown that Nestin is regulated by certain transcription factors to achieve its biological functions [7]. Transcriptional signaling transmitters and activators (STAT) include a family of proteins consisting of the latent cell membrane or intracellular transcription factors, including cellular signaling pathways induced by extrinsic and intrinsic stimuli. Among other activators, Nestin has been shown to be activated by STAT proteins, particularly the STAT3 protein. Moreover, STAT3 activation ultimately leads to the expression or inhibition of several functional genes such as cell proliferation, angiogenesis, inflammation, and apoptosis [8]. Subsequently, STAT3 activation promotes the regulation of signaling pathways directly related to the sex determination region Y) box 2 (SOX2) promoter, leading to Sox2 expression and Nestin expression [9]. Other transcription factors, such as nuclear respiratory factor 2 (Nrf2) are now considered to be key players in the regulation of gene transcription implicated in various cellular functions and cancer development and progression [10].

Studies [11] have demonstrated that Nestin expression can be induced by hypoxia and that the increase in Nestin is regulated in part by hypoxia-inducible factor 1-alpha (HIF-1) and vascular endothelial growth factor (VEGF). Recently, it was demonstrated [12] that severe hypoxia (1% oxygen) enhances the expression of stem cell markers, including Nestin and Sox2 glioma stemlike cells. Although Nestin is expressed in various malignancies, little is known about its role in lung cancer cells. Several studies have shown Nestin expression in nonsmall cell lung cancer (NSCLC), and they all suggest that Nestin is significantly associated with poor differentiation [13]. However, to date, few studies have investigated the mechanistic model of hypoxia-induced Nestin regulation in NSCLC.

RETRACTED

Based on this, we explored how induction of Nestin allows to promote the progression of NSCLC cells by targeting transcription factors Nrf2, STAT3, and SOX2. We first report the following.

## 2. Materials and Methods

### 2.1. Study Population

In this study, 84 cases of NSCLC (cell line A549 and H1299) were randomly selected from our tissue database from patients who had been treated in our Thoracic Department from June 2020 to February 2021. Included patients, had not received any treatment form, chemotherapy or radio chemotherapy. Additional patient information was attained by reviewing their preoperative and perioperative medical records, contact details, and/or written agreements. All participating patients provided a written form consent in accordance with the institution of ethics committee of medical sciences and were approved by the hospital ethical committee. Histopathological studies were performed on the collected samples using hematoxylin and eosin staining, while histological staining was determined according to WHO classification [14]. The size of the tumor and the number and location of metastatic lymph nodes were obtained from the pathology report.

### 2.2. Immunohistochemical Staining and Assessment

Collected sample tissues were immunohistochemically stained with the streptavidin-peroxidase method, and each tissue was deparaffinized, rehydrated, and incubated with fresh 3% methanolic hydrogen peroxide for 15 minutes. The samples were then rinsed with phosphate buffered saline (PBS); antigen was carried out at 100°C in the microwave for 15 minutes in 0.01 mol/L of sodium citrate buffer (pH 6.0). Nonspecific binding was inhibited with normal goat serum for 15 minutes at room temperature then, incubated at 4°C overnight with several antibodies (Table 1). After rinsing with PBS, the slides were then incubated for 10 mins at room temperature with biotin-conjugated secondary antibodies, then incubated with streptavidin-conjugated peroxide solution for 10 minutes. Using 39-diaminobenzidine tetrachloride, sections were stained for 3–5 minutes. Subsequently, tissues were stained with Mayer's hematoxylin, dehydrated, and mounted, negative controls were prepared substituting PBS for primary antibody.

In this study, both cytoplasmic and nucleic staining on Nestin were recorded as positive. Intensity of Nestin expression was scored numerically as, negative = 0, light = 1, moderate = 3, and intense = 3.

### 2.3. Cell Culture

Human nonsmall cell lung cancer (hNSCLS) were cultured in a medium supplemented with 10% (vol/vol) FBS, 100 U/ml penicillin, and 100 *μ*g/ml streptomycin, and incubated at 37°C in humidified environment with 5% CO_2_.

RETRACTED

### 2.4. Western Blotting

Using the RIPA buffer, the Cell lysates were prepared for immunoblotting, then they were supplemented with protease inhibitor cocktail (Roche). After, the lysates were centrifuged at 12,000 × *g* for 10 mins at 4°C for debris removal. Then, the protein concentration was assessed using the BCA Protein assay kit (Thermo). 20 *μ*g of the investigated protein was denatured and resolved using the SDS/PAGE, the target proteins were immunoblotted with antibodies.

### 2.5. Hypoxia Studies

In this study NSCLC cells were plated at 5000 cells/cm^2^ in a 12-well plates and replaced after 24 hrs with preconditioned media from different Oxygen tensions (21% or 1%). At ambient oxygen tension (21%), cells were cultured in a standard humidified incubators at 37°C mixed with 5% CO_2_. At 1% oxygen tension, NSCLC cells were cultured in a humidified incubators at 37°C mixed with 5% CO_2_, 1% Oxygen tension was reduced with supplemented Nitrogen based on default parameters (using the Heracell 1590, Thermo Fisher USA).

### 2.6. PCR Analysis

RNA was purified using the RNeasy Mini Kit (Qiagen), thereafter, samples were transcribed using the using the Qunatitect Reverse Transcription Kit (Qiagen). qPCR NSCLC cell samples were performed, with parameters; 42 cycles of DNA AMPLIFICATION at 94°C for 30 sec, 56–68°C for 30 sec and 72°C for 30 sec.

### 2.7. Statistical Analysis

Data were presented as the mean ± standard deviation (SD), and the error bars represent standard error of the mean. Statistical analysis of means was performed using one-way and two-way ANOVA. Probability level of *P* < 0.05 was considered as statistically significant.

## 3. Results

### 3.1. Basic Clinic Information and Tumor Characteristics

Thirty-three male and twenty-five female patients diagnosed with NSCLC, treated with curative surgical resection were enrolled in this study with a mean age range of 57.5 ± 10 years (range 36–77 years). 29 cases of lung adenocarcinoma, 26 cases of squamous cell carcinoma, and 3 cases of large cell carcinoma were observed amongst the patients. There were 33, 17, and 18 cases with good, moderate, and poor differentiation, respectively, and the observed cases were classified according to the TNM staging system of the International Union Against Cancer (2002), and the cases were classified as stage I (*n* = 33), stage II (*n* = 12), and stage II (*n* = 13) [15]. Thirty-five of these patients had lymph node metastases, and information was obtained for 90% (52/58) of the patients analyzed after 4 years of followup. Other clinical characteristics of the study sample are shown in Table 1.

RETRACTED

### 3.2. Hypoxic Environment Induced Nestin Expression in hLSCs

There was a significant increase in Nestin mRNA expression in hNSCLC at 24 hr postincubation in 1% O_2_ in comparison to cell incubated at 21% O_2_ (Figure 1(a)). An increasing pattern was marked by a significant decrease at 48 hr. Nestin protein levels were significantly greater in 1% O_2_ at both 6 and 24 hrs (Figure 1(b)). Notable increase in Nestin was recorded at 6 and 24 hrs, at which this rise achieved statistical significance (Figure 1(b)). This result suggest that Nestin mRNA and protein levels are increased under hypoxic conditions.

### 3.3. Nestin Expression Is Maintained during hNSCLC Differentiation

To verify the clinicopathological findings of hNSCLC in correlation with nestin expression, cell differentiation was assessed qualitatively. In hNSCLC medium, the increase in staining over time showed a different degree of cell differentiation, consistent with the clinicopathological recordings in Table 1. Statistically, nestin expression was significantly different from controls in hNSCLCs induced to differentiate (Figure 2), but not significantly different in terms of time progression within 10 days.

### 3.4. STAT3 Regulates Nestin Expression via SOX2

To confirm the regulation of the SOX2 promoter by STA3 under Nestin-induced conditions, we introduced STAT3c cells into hNSCLC. These were lysed 48h after transfection, and SOX2 expression was analyzed (Figure 3). We observed that STAT3c successfully induced SOX2 expression in NSCLC cells. Suggesting that SOX2 regulates is an intermediary for STAT3 regulation of Nestin expression.

### 3.5. Nestin Expression Activates the Nrf2 Transcription Factor

The Nrf2 transcription factor is known to regulate the antioxidant defense system. In this study we found that Nestin expression regulates the hNSCLCs through targeting the Nrf2 signaling pathway. To analyze the relationship between Nrf2 and Nestin, NSCLC cells were treated with pivaloyl hydroquinone (tBHQ) and sulfathionine (SF) to analyze the activation of Nrf2. Previous studies have shown that a decrease in Nestin expression decreases the expression of several transcription factors that are targets of Nrf2, such as CAT, GPX1/4, SOD1/2, GCLC/M, HO-1, and NQO1. To investigate this hypothesis, we immunoprecipitated hNSCLC cells with ARE luciferase. Our results showed an increase in Nestin expression induced by hypoxic conditions, which increased the expression of NQO1, GCLM, and HO-1 (Figure 4). The results showed that tBHQ and SF enhanced the protein levels of Nrf2 in both cell lines as compared with the control. Moreover, the transcription of downstream genes were enhanced. These results suggest that the Nestin expression induced by hypoxic conditions regulate the Nrf2 expression.

RETRACTED

### 3.6. Antioxidant Capacity Is Enhanced by Nestin and Nrf2

To determine the role of Nrf2 in Nestin-induced environment in response to oxidative stress, we used overexpression plasmid transfection to alter the expression levels of Nrf2 and Nestin in hNCSLC cells (Figure 5), and we obtained that Nestin maintains redox homeostasis in NSCLC cells by regulating antioxidant capacity. The cells were stimulated with H_2_O_2_ at 48h after transfection. Overexpressed Nrf2 enhanced the resistance of Nestin-knockdown cells to H_2_0_2_-induced toxicity. Furthermore, the suppression of Nrf2 increased the sensitivity of Nestin-overexpressing cell to H_2_O_2_-induced toxicity. Overall, these results showed that overexpressed induced Nestin by hypoxic conditions in association with expression of Nrf2 increase the resistance of Nestin to antioxidative stress.

### 3.7. Nestin, SOX2, STAT3, And Nrf2 Expression in hNSCLC

There were significant differences between primary and metastatic tumor cells throughout the sections, with 12 of 25 (48%) and 3 of 6, STAT3 was not expressed in either cell; whereas 12% and 16% of primary and metastatic tumor cells, respectively, showed positive expression of Nrf2, were positive for Nestin expression, and none of the cells tested positive for SOX2. Interestingly, when Nestin was combined with all the three transcription factors, 40% and 33% of both the primary and metastatic tumor cells tested positive. Proposing a significant relationship of the three in whole section cell growth. Similar trends were observed in the tissue microarray, except the fact SOX2 had increased positive cells, 12.8% and 7.8% in the primary and metastatic tumor cells. Summation the tumor cells that tested positive in different cells in shown in Table 2.

## 4. Discussion

Lung cancer has a poor prognosis and its death rate is the highest among all malignant tumors [5]. Nonsmall cell lung cancer is a common subtype of lung cancer, and platinum-based chemotherapy is still the main treatment for NSCLC patients [16]. In recent years, cell therapy and gene therapy have also been used to treat NSCLC, but their efficacy is still not significant, and the combination of high metastasis rate to other parts of the body in the early stage of NSCLC and the tendency of drug resistance during treatment are clinical characteristics that make the treatment of NSCLC patients unsatisfactory [17]. Despite the rapid development of surgical procedures, radiotherapy, targeted therapies, and immunotherapy, most patients diagnosed with NSCLC have already missed the prime time for treatment, so the search for efficient treatments, the discussion of the evolutionary mechanism and developmental process of NSCLC, and the appropriate interventions for precancerous lesions are the hot topics in the modern research direction of lung cancer treatment [18]. Of particular importance is the significant relationship between hypoxia-induced activation of the Nestin transduction pathway and the formation, drug resistance, recurrence, and poor prognosis of NSCLC [19].

RETRACTED

In the present study, we first confirmed the increased Nestin expression in hNSCLC under hypoxic conditions using two oxygen parameters (O2 at 21% and 1%) associated with increased time. In 1% oxygen, Nestin levels increased at both 6 and 24 hours, peaking at 48 hours, which confirms previous studies that hypoxic conditions induce Nestin expression in cancer tumor cells, in this case lung cancer cells [20]. In support of this phenomenon, hypoxic conditions have been shown to enhance the protumorigenic effects of procollagen lysine hydroxylase 1 (PLOD1) [21]. Studies [22] have shown that Nestin has a common marker for pluripotent stem cells, which is dysregulated in tissue damage and cancer progression. To assess the molecular function of Nestin in lung cancer cells, we analyzed the relationship of Nestin expression with downstream transcription factors, and we demonstrated that Nestin is regulated by STAT3 transcription factor through SOX2 protein. We further investigated the expression relationship of Nestin with another downstream transcription factor and observed that Nestin expression also regulates Nrf2 expression. To understand the induced expression of Nestin and its downstream regulation, we performed whole section and microarray expression analysis on primary and metastatic lung cancer tumor cells. In this regard, we conclude that Nestin regulates the metabolism and viability of human lung cancer cells by combining the regulatory patterns of SOX2, STAT3, and Nrf2. Although previous studies have demonstrated this regulatory pattern, only a few studies have confirmed it in human lung cancer cells [23, 24]. Furthermore, the regulatory mechanism of Nestin still requires further experiments. In this study, we found that Nestin expression levels correlated with the expression of Nrf2 TFs. Studies [25] have recently revealed the role of Nestin in different types of cancer, and they explained that Nestin, as a marker of microvascular density, is a reliable prognostic factor for neoplastic malignancies. The study [26] also reported that SOX2 is a signal transducer and activator of STAT3 and Nestin in a model of inhibition of glioblastoma multiforme (GMB). In their study [27], they showed that Nestin and SOX2 were coexpressed in human melanoma tissues, which subsequently triggered STAT3 expression. This result raises the possibility that Nestin/SOX2/STAT3/Nrf2 may confer greater clinical virulence, which is consistent with previous studies [28, 29].

RETRACTED

However, our study has some shortcomings; the prognostic value of inducible Nestin in lung cancer was not estimated in several clinical samples, and only a few patients and their cell samples were included in this study. In addition, the follow-up period was not extended.

## 5. Conclusion

In summary, we conclude that hypoxia-induced Nestin targets STAT3, SOX2, and Nrf2, induces their expression, and leads to increased metastatic spread in hNSCLC. Although our study has some limitations, it also provides some clinical basis that the goal of saving the lives of NSCLC patients and prolonging their survival will eventually be achieved.

## Figures and Tables

**Figure 1:** Hypoxia conditions promote nestin expression in hNSCLC. *Note*. (a) qPCR analysis of Nestin expression at 6, 24, and 48 hr, cultured 21% and 0% O_2_; (*P* < 0.05). (b) Quantification of Nestin protein expression in hNSCLC cultured at 21% and 0% O_2._ Bars represent mean protein expression normalized.

**Figure 2:** Effects of time in human nonsmall lung cancer media on Nestin expression. *Note*. Bars represent mean nestin expression normalized.

**Figure 3:** Nestin regulation analysis by the STAT3 protein expression through an intermediate SOX2. *Note*. Mean protein expression is represented by blue and orange bars in the graph, shows an 1% and 21% Oxygen content in both Nestin-induced and Nestin-knockdown environments.

**Figure 4:** Luciferase assay to investigate the effect of Nestin on cellular antioxidant activity mediated in the Nrf2-ARE pathway. Note: hNSCLS cells with and without Nestin knockdown were transfected with ARE reporter gene plasmid. Results showed a fold change of luciferase activity.

**Figure 5:** Nestin and Nrf2 increase the resistance to antioxidant capacity. Note: Statistical evaluation of overexpressed Nestin and Nrf2 A549 cells. Bars represent percentage of apoptotic cells, data is defined as the means ± SD, *P* < 0.05 considered statistically significant.

**Table 1:** Relationship of the Nestin expression in hNSCLC with clinical and pathological factors.

	Patients	NESTIN-low, *n* (%)	NESTIN-high, *n* (%)	*P* (value)
Sex				
Female	25	17 (54.0)	8 (46.0)	0.548
Male	33	18 (43.9)	15 (56.1)	

Age (y)				
≤60	36	20 (44.7)	16 (55.3)	0.298
>60	22	12 (58.7)	10 (41.3)	

Smoking				
Yes	34	28 (60.7)	6 (39.3)	0.155
No	24	14 (33.3)	10 (66.7)	

Diffrentitian				
Good	23	15 (67.3)	8 (32.7)	0.047
Moderate	17	8 (34.5)	9 (63.5)	
Poor	18	12 (67.4)	4 (32.6)	

TNM stage				
I	33	15 (61.7)	18 (38.3)	0.189
II	12	7 (56.0)	5 (43.0)	
III	13	6 (45.9)	7 (56.1)	

Histology				
Adenocarcinoma	29	19 (53.8)	10 (46.2)	0.003
Squamous cell carcinoma	26	13 (50.3)	13 (49.7)	
Large cell carinoma	3	1 (50.0)	2 (50.0)	

Lymph node metastasis				
N0	23	14 (72.2)	9 (27.8)	0.009
N1	20	9 (61.3)	11 (38.7)	
N2	15	10 (78.9)	5 (21.1)	

MVD expression				
High	30	19 (64.9)	11 (35.1)	0.22
Low	22	14 (56.9)	8 (43.1)	

Lvd expresssion				
High	34	20 (48.3)	14 (51.7)	0.874
Low	24	13 (73.6)	9 (26.4)	

VEGF expression				
High	29	15 (61.9)	14 (38.1)	0.754
Low	29	18 (40.0)	11 (60.0)	

COX-2 expression				
High	28	17 (68.3)	11 (31.7)	0.269
Low	30	22 (62.0)	8 (38.0)	

RETRACTED

**Table 2:** Nestin, Sox2, STA3, and Nrf2 immunoreactivity in human nonsmall cell lung cancer.

	Whole section		Tissue microarrays	
	Primary (%)	Metastitic (%)	Primary (%)	Metastic (%)
NESTIN	12 (48)	3 (50)	17 (16.8)	5 (13.2)
SOX2	0	0	13 (12.8)	3 (7.8)
NRF2	3 (12)	1 (16)	0	3 (7.8)
STAT3	0	0	15 (14.8)	4 (10.5)
COMBINED	10 (40)	2 (33)	45 (44.5)	22 (57.9)
NEITHER	0	0	11 (10.8)	0
TOTAL	25	6	101	38

## Data Availability

The data used to support the findings of this study are available from the corresponding author upon request.

## References

[1] Sung H., Ferlay J., Siegel R. L. (2021). Global cancer statistics 2020: GLOBOCAN estimates of incidence and mortality worldwide for 36 cancers in 185 countries. *CA: A Cancer Journal for Clinicians*.

[2] Agliano A., Calvo A., Box C. (2017). The challenge of targeting cancer stem cells to halt metastasis. *Seminars in Cancer Biology*.

[3] Arnold C. R., Mangesius J., Skvortsova I. I., Ganswindt U. (2020). The role of cancer stem cells in radiation resistance. *Frontiers in Oncology*.

[4] Sone K., Maeno K., Masaki A. (2020). Nestin expression affects resistance to chemotherapy and clinical outcome in small cell lung cancer. *Frontiers in Oncology*.

[5] Jaramillo-Rangel G., Chávez-Briones M.-d.-L., Ancer-Arellano A., Ortega-Martínez M. (2021). Nestin-expressing cells in the lung: the bad and the good parts. *Cells*.

[6] Das T., Kamle A., Kumar A., Chakravarty S. (2021). Hypoxia induced sex-difference in zebrafish brain proteome profile reveals the crucial role of H3K9me3 in recovery from acute hypoxia. *Frontiers in Genetics*.

[7] Wong A., Ghassemi E., Yellowley C. E. (2014). Nestin expression in mesenchymal stromal cells: regulation by hypoxia and osteogenesis. *BMC Veterinary Research*.

[8] He S., Lin J., Lin L., Xu Y., Feng J. (2018). Shikonin-mediated inhibition of nestin affects hypoxia-induced proliferation of pulmonary artery smooth muscle cells. *Molecular Medicine Reports*.

RETRACTED

[9] Nishikawa M., Inoue A., Ohnishi T. (2021). Hypoxia-induced phenotypic transition from highly invasive to less invasive tumors in glioma stem-like cells: significance of CD44 and osteopontin as therapeutic targets in glioblastoma. *Translational Oncology*.

[10] Chen Z., Wang T., Luo H. (2010). Expression of nestin in lymph node metastasis and lymphangiogenesis in non-small cell lung cancer patients. *Human Pathology*.

[11] Lin Y., Song Z., Xi Z. (2021). The anticancer potency of artemisinin and its derivatives. *SPR*.

[12] Barta J. A., Powell C. A., Wisnivesky J. P. (2019). Global epidemiology of lung cancer. *Annals of Global Health*.

[13] Travis W. D., Brambilla E., Nicholson A. G. (2015). The 2015 world health organization classification of lung tumors: impact of genetic, clinical and radiologic advances since the 2004 classification. *Journal of Thoracic Oncology*.

[14] Castrogiovanni P., Mazzone V., Imbesi R. (2011). Immunolocalization of HB-EGF in human skin by streptavidin-peroxidase (HRP) conjugate method. *International Journal of Morphology*.

[15] Greene F. L., Balch C. M., Fleming I. D. (2002). *AJCC Cancer Staging Handbook: TNM Classification of Malignant Tumors*.

[16] Ma Q., He X. (2012). Molecular basis of electrophilic and oxidative defense: promises and perils of Nrf2. *Pharmacological Reviews*.

[17] Wang J., Cai J., Huang Y. (2016). Nestin regulates proliferation and invasion of gastrointestinal stromal tumor cells by altering mitochondrial dynamics. *Oncogene*.

[18] Zhang C. C., Sadek H. A. (2014). Hypoxia and metabolic properties of hematopoietic stem cells. *Antioxidants and Redox Signaling*.

[19] Liu F., Zhang Y., Lu M. (2017). Nestin servers as a promising prognostic biomarker in non-small cell lung cancer. *American Journal of Tourism Research*.

[20] Wang Z., Shi Y., Ying C., Jiang Y., Hu J. (2021). Hypoxia-induced PLOD1 overexpression contributes to the malignant phenotype of glioblastoma via NF-*κ*B signaling. *Oncogene*.

[21] Jiang M. H., Cai B., Tuo Y. (2014). Characterization of Nestin-positive stem Leydig cells as a potential source for the treatment of testicular Leydig cell dysfunction. *Cell Research*.

[22] Zhang C., Mukherjee S., Tucker‐Burden C. (2017). TRIM 8 regulates stemness in glioblastoma through PIAS 3‐STAT 3. *Molecular oncology*.

[23] Fan Y., Xue W., Schachner M., Zhao W. (2018). Honokiol eliminates glioma/glioblastoma stem cell-like cells via JAK-STAT3 signaling and inhibits tumor progression by targeting epidermal growth factor receptor. *Cancers*.

RETRACTED

[24] Ejaz H., Saharan Q. M., Ashiq S. (2021). Elimination of heavy metals and pesticides from wastewater by using Bagasse Fly Ash. *SPR*.

[25] Wang J., Lu Q., Cai J. (2019). Nestin regulates cellular redox homeostasis in lung cancer through the Keap1–Nrf2 feedback loop. *Nature Communications*.

[26] Szymańska-Chabowska A., Świątkowski F., Jankowska-Polańska B., Mazur G., Chabowski M. (2021). Nestin expression as a diagnostic and prognostic marker in colorectal cancer and other tumors. Clinical medicine insights. *Oncology*.

[27] Chuang H.-Y., Su Y.-k., Liu H.-W. (2019). Preclinical evidence of STAT3 inhibitor pacritinib overcoming temozolomide resistance via downregulating miR-21-enriched exosomes from M2 glioblastoma-associated macrophages. *Journal of Clinical Medicine*.

[28] Zhang S., Cui W. (2014). Sox2, a key factor in the regulation of pluripotency and neural differentiation. *World Journal of Stem Cells*.

[29] Yuan X. F., Wen X., Ling Y., Li M. L. (2021). FXR mediated bile acid signal to advance the study of cirrhosis of the liver regeneration. *SPR*.

